# Efficacy of *Bifidobacterium* Triple Viable Enteric-Coated Capsules Combined with Enteral Nutrition on Patients with Chronic Critical Illness and Influence on Immune and Coagulation Function

This article has been retracted.

**DOI:** 10.1155/2021/3718255

**Published:** 2021-10-15

**Authors:** Wei Wang, Hui Zhang, Wenjuan Huang

**Affiliations:** ^1^Department of ICU, Zhuji People's Hospital, Zhuji 311800, Zhejiang, China; ^2^Department of EICU, The First People's Hospital of Yongkang, Yongkang 321302, Zhejiang, China

## Abstract

**Objective:**

To investigate the efficacy of enteric-coated *Bifidobacterium* triple viable capsules combined with enteral nutrition in the treatment of patients with chronic critical illness (CCI) and their effects on the immune and coagulation function of patients.

**Methods:**

106 CCI patients admitted to the intensive care unit of our hospital from December 2018 to March 2020 were selected as the research objects, and they were randomly divided into the control group (*n* = 53) and the observation group (*n* = 53). The control group was given symptomatic treatment, etiological treatment, clinical nursing, enteral nutrition support, and other conventional treatment methods according to the patient's condition. On this basis, the observation group was treated with enteric-coated *Bifidobacterium* triple viable capsules, and both groups were treated for 14 days. All patients were followed up for 3 months after treatment, and their death/cure prognosis was recorded. The acute physiological and chronic health (APACHE II) scoring system was used to evaluate the acute physiological and chronic health status of the two groups before and after treatment, and the organs of the patients were scored with sepsis-related organ failure assessment (SOFA) score. T lymphocyte subsets (CD3+, CD4+, CD8+, and CD4+/CD8+), prothrombin time (PT), activated partial thrombin time (APTT), fibrinogen (FIB), and D-dimer (DD) were measured before and after treatment.

**Results:**

The cure rate of the observation group was slightly higher than that of the control group, and the mortality rate was slightly lower than that of the control group, but the difference was not statistically significant (*P* < 0.05). After treatment, the APACHE II and SOFA scores of the two groups were lower than before treatment, and the APACHE II and SOFA scores of the observation group were lower than those of the control group, and the differences were both statistically significant (*P* < 0.05). After treatment, the levels of CD3+, CD4+, and CD4+/CD8+ in the two groups were higher than those before treatment, and the levels of CD8+ were lower than before treatment. The CD3+, CD4+, and CD4+/CD8+ levels of the observation group were higher than those of the control group, and the CD8+ levels were lower than the control group, and the differences were both statistically significant (*P* < 0.05). After treatment, the PT and APTT levels of the two groups of patients were higher than those before treatment, and the levels of FIB and DD were lower than those before treatment. The PT and APTT levels of the observation group were higher than those of the control group, and the FIB and DD levels were lower than those of the control group, and the differences were both statistically significant (*P* < 0.05).

**Conclusion:**

The combination of enteric-coated *Bifidobacterium* triple viable capsules and enteral nutrition for CCI has high cure rate, which can not only improve the patients' physiological health status and organ dysfunction but also effectively improve the patients' immune and coagulation function, which is worthy of promotion.

## 1. Introduction

Chronic critical illness (CCI) refers to critically ill patients who have passed the acute risk period of the disease, but still have organ dysfunction, and need to rely on mechanical ventilation, blood filtration, and other life support and care for a long time [1, 2]. CCI patients usually have internal environmental disorders and persistent dysfunction, which trigger a series of syndromes such as continuous inflammatory response, immunosuppression, and coagulation dysfunction. In severe cases, it can even lead to death and seriously endanger the patient's life safety [3, 4]. The gastrointestinal tract is not only a simple digestion and absorption organ but also an important immune organ, and the intestinal flora can provide nutrition for the body, regulate metabolism, regulate intestinal epithelial development, and induce innate immunity. Imbalance of intestinal flora can lead to intestines abnormal tract barrier function; microbial-mediated inflammation can directly induce or aggravate the abnormal immune function and coagulation function of patients, which seriously affects the prognosis of patients [5, 6]. Therefore, improving the immune and coagulation function of the patient's intestinal tract is extremely important for the treatment of CCI. The microecological regulator is a medicine prepared according to the principle of microecology, which can adjust the balance of intestinal flora, build the balance of intestinal microecology, improve the immune function, and improve the inflammatory response in the body. Nutritional support is an indispensable part of the treatment of CCI patients. Since most patients cannot eat by mouth, enteral nutrition has become the first choice for nutritional support treatment [7, 8]. The purpose of this study was to investigate the efficacy of microecological modulators (*Bifidobacterium* triple viable enteric-coated capsules) combined with enteral nutrition in the treatment of CCI patients and its effect on the immune and coagulation function of patients. The specific report is as follows.

## 2. Materials and Methods

### 2.1. General Information

A total of 106 CCI patients admitted to the intensive care unit of our hospital from December 2018 to March 2020 were selected as the study subjects, including 62 males and 44 females, aged 31–72 years old, with an average age of (53.84 ± 10.38) years old. Inclusion criteria: all patients were diagnosed as CCI patients after clinical diagnosis; complete clinical data; those who did not fall off during the follow-up period. Exclusion criteria: patients with malignant tumors; those who are pregnant and malnourished; people with congenital immune dysfunction; serious intolerance during treatment; those with poor compliance; severe history or injury of the digestive tract; tumor patients; death during treatment. The 106 patients were divided into a control group and an observation group using a random number table method, with 53 cases in each group. Among them, there were 32 males in the control group and 21 females, aged 33–72 years old, with an average age of (54.02 ± 10.78) years old. In the observation group, there were 30 males and 23 females, aged 31–70 years old, with an average age of (53.68 ± 10.22) years old. There was no statistical difference between the two groups of gender and age in general data (*P* > 0.05), and they were comparable. This study was approved by the ethics committee of our hospital, and the patients and their family members gave informed consent and signed an informed consent form.

### 2.2. Research Methods

The control group was given symptomatic treatment, etiological treatment, clinical nursing, enteral nutrition support, and other conventional treatment methods according to the patient's condition. On this basis, the observation group was given a microecological regulator for treatment. The microecological regulator used *Bifidobacterium* triple viable enteric-coated capsules (Jincheng Haisi Pharmaceutical Co., Ltd., National Medicine Standard S19993065, 210 mg *∗* 24 capsules), 420 mg each time, 3 times a day. Treatment lasts for 14 days.

All patients were followed up for 3 months after treatment, and their death/cure prognosis was recorded. The acute physiology and chronic health evaluation (APACHE II) score system [9] was used to evaluate the acute physiology and chronic health status of the two groups before and after treatment. The higher the score means the more severe the illness. Before and after treatment, the organ failure (sepsis-related organ failure assessment, SOFA) score [10] was used to score the patient's organs. The higher the score means the more severe the disease. Before and after treatment, fasting venous blood was taken from the two groups of patients, immunofluorescence flow cytometry was used to determine the T lymphocyte subsets (CD3+, CD4+, CD8+, CD4+/CD8+), and the automatic blood coagulometer was used to detect and compare the thrombin of the two groups. Prothrombin time (PT), activated partial thromboplastin time (APTT), fibrinogen (FIB) level, and D-dimer (DD) level, the serum albumin (ALB), prealbumin (PA), transferrin (TRF), and hemoglobin (Hb) levels of the two groups were determined before and after treatment.

### 2.3. Statistical Methods

The results of this experiment were statistically analyzed by SPSS 20.0 (SPSS Co., Ltd., Chicago, USA). Count data were expressed by (rate), and the chi-square test was used for their comparison between groups. Measurement data were expressed by (mean ± standard deviation), and the *t*-test was used for their comparison between groups. *P* < 0.05 indicates that the difference is statistically significant.

## 3. Results

### 3.1. Comparison of the Prognosis of the Two Groups of Patients

During the treatment period, there were 3 patients in the control group and 2 patients in the observation group. The family members signed and agreed to terminate or transfer the treatment. During the follow-up process after treatment, 45 cases (90.00%) in the control group were cured and 5 cases (10.00%) died. In the observation group, 49 cases (96.08%) were cured and 2 cases (3.92%) died. The cure rate of the observation group was slightly higher than that of the control group, and the mortality rate was slightly lower than that of the control group, but the difference was not statistically significant (*P* > 0.05), as given in Table 1.

### 3.2. Comparison of APACHE II and SOFA Scores between the Two Groups

After treatment, the APACHE II and SOFA scores of the two groups were lower than before treatment, and the APACHE II and SOFA scores of the observation group were lower than those of the control group. The differences were statistically significant (*P* < 0.05), as given in Table 2.

### 3.3. Comparison of the Immune Function of the Two Groups of Patients

After treatment, the levels of CD3+, CD4+, and CD4+/CD8+ in the two groups were higher than those before treatment, the level of CD8+ was lower than before treatment, and the levels of CD3+, CD4+, and CD4+/CD8+ in the observation group were higher than those in the control group. The CD8+ level was lower than that of the control group, and the difference was statistically significant (*P* < 0.05), as shown in Figure 1.

### 3.4. Comparison of the Coagulation Function of the Two Groups of Patients

After treatment, the PT and APTT levels of the two groups of patients were higher than before treatment, and the levels of FIB and D-D were lower than before treatment. The PT and APTT levels of the observation group were higher than those of the control group, and the FIB and D-D levels were lower than those of the control group. The differences were statistically significant (*P* < 0.05), as shown in Figure 2.

### 3.5. Comparison of Nutritional Status between the Two Groups

After treatment, the serum ALB, PA, TRF, and Hb levels of the two groups were significantly lower than before treatment, and the serum ALB, PA, TRF, and Hb levels of the observation group were significantly higher than those of the control group (*P* < 0.05), as shown in Figure 3.

## 4. Discussion

CCI is a specific stage in the development and outcome of critical illness, often accompanied by severe malnutrition, immune disorders, and coagulation dysfunction [11, 12]. Therefore, while giving patients nutritional support treatment, it is also necessary to deal with the patient's immune and coagulation abnormalities. Intestinal microbes play an important role in human health. They form a symbiotic relationship with the host during the evolution process and play an important role in regulating the host's digestion and absorption, metabolism, and immune response [12, 13]. *Bifidobacterium* triple viable enteric-coated capsules are probiotic preparations composed of *Bifidobacterium longum*, *Lactobacillus acidophilus*, and *Enterococcus faecalis*. Probiotics are active microorganisms, which can improve the ecological balance of the host's intestinal flora, thereby, adjusting the intestinal flora, improving the intestinal microecology of the patient, and improving the prognosis [14, 15].

The results of this study showed that during the follow-up after treatment, 45 cases (90.00%) were cured and 5 cases (10.00%) died in the control group. In the observation group, 49 cases (96.08%) were cured and 2 cases (3.92%) died. The observation group's cure rate was slightly higher than that of the control group, and the mortality rate was slightly lower than that of the control group. The results of the study showed that after treatment, the APACHE II and SOFA scores of the two groups were lower than those before treatment, and the APACHE II and SOFA scores of the observation group were lower than those of the control group. It shows that the microecological regulator combined with enteral nutrition therapy can improve the patient's physical health and organ dysfunction and has a certain effect on improving the cure rate and reducing the mortality rate. Analysis of the reason is that enteral nutrition support therapy not only provides sufficient nutrients to patients but also regulates internal environmental disorders and immune function, enhances the body's resistance to diseases, and thus facilitates the recovery of patients. When combined with a microecological regulator, the probiotics in the agent can adhere to the epithelial cells of the intestinal mucosa, which can fully adjust the balance of the intestinal flora, promote the digestion and absorption of food, and reduce the absorption of toxins and metabolites. It is more conducive to the prognosis of patients [16, 17].

The results of this study showed that after treatment, the levels of CD3+, CD4+, and CD4+/CD8+ in the two groups were higher than those before treatment, the levels of CD8+ were lower than before treatment, and the levels of CD3+, CD4+, and CD4+/CD8+ in the observation group were higher than those in the control group. Lower than the control group, it shows that the combination of microecological modulator and enteral nutrition therapy can better improve the immune function of patients. The reason is that after probiotics enter the intestine, they can not only effectively ensure the balance of intestinal microbes but also restore intestinal peristalsis, reduce intestinal mucosal epithelial cell apoptosis, protect the barrier function of intestinal mucosa, and inhibit local inflammation of intestinal mucosa. Enhance the immune function of patients [18, 19]. The results of the study showed that after treatment, the levels of PT and APTT of the two groups were higher than those before treatment, and the levels of FIB and DD were lower than those before treatment. The PT and APTT levels of the observation group were higher than those of the control group, and the levels of FIB and DD were lower than those before treatment. Control group shows that the combination of microecological modulator and enteral nutrition therapy can improve the blood coagulation function of patients. The reason is that the inflammatory response mediated by toxins or pathogenic microorganisms can directly induce or aggravate abnormal blood coagulation. The enzymes produced by probiotics, their metabolites, and cell wall components are good antidotes. Reduce the intestinal absorption of toxins and metabolites, which is beneficial to the recovery of the patient's blood coagulation function [20, 21]. The results of this study showed that after treatment, the serum ALB, PA, TRF, and Hb levels in the two groups were significantly lower than before treatment, and the serum ALB, PA, TRF, and Hb levels in the observation group were significantly higher than those in the control group. These results indicate that *Bifidobacterium* triple viable enteral capsule combined with enteral nutrition therapy can effectively restore the nutritional status of CCI patients.

In summary, the combination of *Bifidobacterium* triple live bacteria enteric-coated capsules combined with enteral nutrition has a higher cure rate for CCI. It not only improves the patient's physical health and organ dysfunction but also effectively improves the patient's immune and coagulation function. It is worthy of promotion for clinical usage.

## Figures and Tables

**Figure 1:** Comparison of the immune function of the two groups of patients. Note: compared with before treatment, ^*∗*^*P* < 0.05; compared with the control group, ^#^*P* < 0.05.

**Figure 2:** Comparison of the coagulation function of the two groups of patients. Note: compared with before treatment, ^*∗*^*P* < 0.05; compared with the control group, ^#^*P* < 0.05.

**Figure 3:** Comparison of nutritional status between the two groups. Note: compared with before treatment, ^*∗*^*P* < 0.05; compared with the control group, ^#^*P* < 0.05.

**Table 1:** Comparison of the prognosis of the two groups of patients.

Group	Cure	Dead
Control group (*n* = 50)	45 (90.00%)	5 (10.00%)
Observation group (*n* = 51)	49 (96.08%)	2 (3.92%)
*χ* ^2^ value	1.446	
*P* value	0.229	

**Table 2:** Comparison of APACHE II and SOFA scores between the two groups of patients.

Group	APACHE II score (score)		SOFA score (score)	
	Before treatment	After treatment	Before treatment	After treatment
Control group (*n* = 50)	20.15 ± 2.58	14.21 ± 1.36^*∗*^	10.52 ± 1.26	7.26 ± 0.84^*∗*^
Observation group (*n* = 51)	20.01 ± 2.18	10.08 ± 0.95^*∗*^	10.43 ± 1.41	4.35 ± 1.21^*∗*^
*t* value	0.302	18.124	0.346	14.382
*P* value	0.763	<0.001	0.729	<0.001

*Note.* Compared with this group before treatment, ^*∗*^*P* < 0.05.

## Data Availability

The data used and/or analyzed during the current study are available from the corresponding author upon request.
